The article "Investigating the Effect of Hydroalcoholic Extract of Licorice Root to Prevent Ovariectomy-Mediated Complications" was published in 2022. Journal: Biomed Res Int.

# Investigating the Effect of Hydroalcoholic Extract of Licorice Root to Prevent Ovariectomy-Mediated Complications

**DOI:** 10.1155/2022/7879432

**Published:** 2022-08-10

**Authors:** Nader Tanideh, Zahra Zareian, Reza Hosseinpour, Romina Tanideh, Farhad Koohpeyma, Omid Koohi-Hosseinabadi, Golsa Shekarkhar, Cambyz Irajie, Maryam Mojahed Taghi, Mohammad Javad Yavari Barhaghtalab, Aida Iraji

**Affiliations:** ^1^Stem Cells Technology Research Center, Shiraz University of Medical Sciences, Shiraz, Iran; ^2^Department of Pharmacology, School of Medicine, Shiraz University of Medical Sciences, Shiraz, Iran; ^3^Student Research Committee, Shiraz University of Medical Sciences, Shiraz, Iran; ^4^Department of General Surgery, Shahid Jalil Hospital, School of Medicine, Yasuj University of Medical Sciences, Yasuj, Iran; ^5^Endocrinology and Metabolism Research Center, Shiraz University of Medical Sciences, Shiraz, Iran; ^6^Laparoscopy Research Center, Shiraz University of Medical Sciences, Shiraz, Iran; ^7^Central Research Laboratory, Shiraz University of Medical Sciences, Shiraz, Iran; ^8^Department of Pathology, Shiraz University of Medical Sciences, School of Medicine, Shiraz, Iran; ^9^Department of Medical Biotechnology, School of Advanced Medical Sciences and Technologies, Shiraz University of Medical Sciences, Shiraz, Iran

## Abstract

**Introduction:**

The importance of women's health and the quality of life after menopause is a critical issue. To prevent disability and menopause complications as well as avoid the side effects of hormone replacement therapy (HRT), in this study, licorice hydroalcoholic extract (*Glycyrrhiza uralensis* roots) was evaluated as a natural remedy.

**Methods:**

Seventy-two female Sprague-Dawley rats were divided into six groups: control group, Sham-operated group, Glycyrrhiza (Gly) 30% group, and ovariectomized group as well as two ovariectomized groups treated with Gly 10% and Gly 30%. Normal saline and different treatments were administered orally for 8 weeks. At the end of the study, calcium, alkaline phosphatase, estrogen, and progesterone levels in the ovariectomized rats were determined. Moreover, the stereological and histopathological changes in uterine tissue in all groups were determined. Phytochemical analyses were also performed to determine the total phenolic content and antioxidant potential of the extract.

**Result:**

The hydroalcoholic extract of licorice root exhibited considerable effect to improve calcium, estrogen, and progesterone levels in the ovariectomized rats. Also, hydroalcoholic extract of licorice root successfully decreases the amount of alkaline phosphatase (ALP) level. The stereological and histopathological findings confirmed the therapeutic potential of this extract. The considerable effects of hydroalcoholic extract of licorice root could be due to high amounts of phytoestrogens with similar estrogen-like structures. Considerable total phenolic content and antioxidant activity were also seen in licorice root extract.

**Conclusion:**

Hydroalcoholic extract of licorice root due to containing high amounts of phytoestrogens with similar chemical structures to estradiol notably improves biochemical parameters as well as stereological and histopathological markers of uterine tissues in ovariectomy rats, so it could be a potential agent for prevention and/or treatment as hormone replacement therapy in healthy middle-aged and/or older women.

## 1. Introduction

The high frequency of age-related diseases and their complications often differ between the sexes promoting researchers targeting them through noninvasive methods. In recent years, the emergence of specific diseases, which undoubtedly contribute to disparate life expectancies, has had significant impacts on the quality of life and health care costs [1–3]. Specifically, menopause is a natural physiological process in older women that are associated with reduced estrogen production and results in an increased risk of diabetes, obesity, stroke, and osteoporosis as well as genitourinary and sexual dysfunction [4–7]. According to the North American Menopause Society (NAMS), around 6000 US women transition to menopause each day [8]. It has been estimated that women will be spending more time in a postmenopausal state than before. Estrogens as one of the most important sexual hormones are mainly produced in the ovarian internal theca cells through the conversion of cholesterol to androstenedione or testosterone, being subsequently aromatized to estrone and estradiol in granulosa cells [9–11]. Sexual hormones, such as estrogen and progesterone, modulate skeletal homeostasis *via* effects on osteocytes and osteoblasts, reducing bone resorption, remodeling, and supporting the maintenance of bone formation [12, 13]. In addition to bothersome symptoms and complications mentioned above, long-term postmenopausal genitourinary increases the risk of cognitive decline as well as cancer especially breast cancer [14].

In recent years, the use of natural remedies has increased mainly in chronic diseases due to the reduced intake and the long period of consumption of synthetic drugs and hormone therapy. The licorice root (*Glycyrrhiza glabra L*.) belongs to the Fabaceae family and is widely used as a sweetening and flavoring agent in food industries as well as in various clinical applications [15]. Licorice extends from southern Europe to central Asia cultivated on a large scale in Belgium, Britain, France, Germany, and Italy. The plant wildly grows in various countries, including China, Turkey, and Iran [16]. Licorice root has been widely used in traditional global and Persian medicine including acute infections, respiratory infections, strep throat, and ulcer healing, as well as kidney and urinary system diseases [17, 18]. The pharmacological effects of licorice are attributed to its various metabolites and natural products. Major bioactive component of licorice root extract, isolated by now, includes more than 50 triterpenoids, around 200 individual phenolic compounds, and hundreds of polysaccharides and amino acids [19–21].

Ovariectomy (OVX) has been accepted as a standard procedure to investigate monophenolase and its complications in which the surgical procedure is performed to remove the ovary with surgery [22]. This procedure deprives the body of the hormones, such as estrogen and progesterone, produced in the ovaries, leading to OVX complications. It was shown that the OVX in female rats is an approved ideal model to assess complications and possible therapeutic approaches related to menopause.

The present study aimed to evaluate the effects of hydroalcoholic extract of licorice root on the lipid profiles, biochemical, and hormonal indexes in serum of the OVX animal model. Also histopathological and stereological assessments on the uterine tissue were performed. It was hypothesized that licorice could be an alternative approach to treating or preventing many age-related diseases.

## 2. Materials and Methods

### 2.1. Ethical Statement

All the procedures were in agreement with the guidelines of the Committee on Research Ethics of the Shiraz University of Medical Sciences (IR.SUMS.MED.REC.1399.304) and the international standards and national legislation on animal care and the Animal Research Reporting In vivo Experiments (ARRIVE) guidelines. Experimental research on the plant was under international legislation and guidelines of the Pharmacognosy Department of Shiraz University of Medical Sciences, Shiraz, Iran.

### 2.2. Plant Extract

The licorice roots were bought from the local market in Shiraz, Iran, and the species were identified by a botanist. Surface cleaned roots were shade-dried and macerated with 70% ethanol : water at room temperature for 1 day. The maceration step was repeated 3-4 times. The obtained extract was filtrated and concentrated in a vacuum using a rotary flash evaporator. The extract was stored at 20°C for later use. The yield was around 15% w/w.

### 2.3. Determination of the Total Phenolic Content of Hydroalcoholic Extract of Licorice Root

The total phenolic content (TPC) of the hydroalcoholic extract of licorice root was evaluated according to the modified Folin-Ciocalteu spectrophotometric method described previously. An aliquot of 5 *µ*l solution of the extract was added to 160 *µ*l water and 10 µl Folin-Ciocalteu agents. The mixture was mixed well for 8 minutes. To this solution, 30 *µ*l of a 25% sodium carbonate solution was added. The above solution was further incubated at room temperature for 2 hours in the dark and its absorbance was measured at 765 nm against the blank using an ultraviolet-visible spectrophotometer. The same procedure was repeated for the standard solution of gallic acid and the calibration standard curve was construed. The measurement was compared to a standard curve prepared with a gallic acid solution. The concentration of the total phenols was expressed as milligrams of gallic acid equivalents per gram of dry extract (mg of GAE/g of dry extract) [23–25].

### 2.4. Determination of the Antioxidant Activity of Hydroalcoholic Extract of Licorice Root

The antioxidant capacity of the extract was calculated using a 2, 2-diphenyl-1-picrylhy-drazyl (DPPH) assay. DPPH is characterized as a stable radical containing the delocalization electron with a deep violet color. The odd electron of DPPH absorbed a hydrogen atom from antioxidants and the reduction of violet color took place. A stock solution of DPPH (110 *μ*M) was prepared freshly by dissolving the appropriate amount in methanol. A volume of 20 *µ*l of different concentrations of the sample extract or standard quercetin and 180 *µ*l of methanol (with or without DPPH) were mixed in a 96-well plate at 25°C temperature for 30 min. The absorbance was measured at 517 nm against methanol as blank. Values were expressed as the mean standard error of the mean (SEM) of triplicate experiments [25–27].

### 2.5. Housing and Selection of Animals

Seventy-two female Sprague-Dawley rats, aged 6 months, weighing between 200 ± 20 g were purchased from the Laboratory Animals Center, Shiraz University of Medical Sciences, Shiraz, Iran. All rats were maintained on a 12-hour light-dark cycle at 25°C, with humidity between 60 ± 10%. The rats were housed in polyethylene cages and given free access to standard rat chow pellets and water during the acclimatization period.

### 2.6. Experimental Design

Rats were divided into six groups, randomly each containing 12 animals:

Control group: received 1 ml of normal saline once a day, orally.

Sham-operated group: received 1 ml of normal saline once a day, orally.

Gly 30% group: received 30 mg/kg of hydroalcoholic extract of licorice root once a day, orally.

Group OVX as a negative control: OVX rats received 1 ml of normal saline once a day, orally.

Groups OVX+ Gly 10%: OVX rats received 10 mg/kg of hydroalcoholic extract of licorice root once a day, orally.

Groups OVX+ Gly 30%: OVX rats received 30 mg/kg of hydroalcoholic extract of licorice root once a day, orally.

Daily oral administration of the vehicle or hydroalcoholic extract of licorice root was performed for 8 weeks after inducing OVX.

### 2.7. Ovariectomy and Sham Surgery Procedure

Rats were anesthetized with xylazine 2% (10 mg/kg) and ketamine 10% (100 mg/kg). The skin was shaved off, and bilateral dorsolateral incisions were carried out through the skin. After ligation of the uterine horn through a midline longitudinal incision, both ovaries were surgically removed in all the groups, except for the control and Gly 30% groups. The Sham-operated rats had their ventral incision and the manipulation of ovaries was performed without excising them [28].

### 2.8. Biochemical Investigations

Enzymatic colorimetric methods were performed after eight weeks to determine the effects of licorice root hydroalcoholic extract on calcium and alkaline phosphatase (ALP) levels. In this regard, blood samples were collected into the chilled nonheparinized tubes, left for clotting, and then centrifuged at 3500 rpm at 4°C for 20 min to prepare the serum [29]. Estrogen and progesterone levels were also calculated by enzyme-linked immunosorbent assay (ELISA) biochemical technique [25].

### 2.9. Stereological Measurements

The Cavalieri method was applied to estimate the total volume of the uterine horn. To estimate the volume, the uterine horn was divided into 8 to 12 parallel sections with a specified distance (t). After tissue processing, the sections were placed in paraffin blocks. Serial 5 *μ*m thick sections were taken using a microtome and stained with Hematoxylin and Eosin (H&E) (Merck company, Germany) method.

A point grid was used to calculate the slice area, which was completely randomized to the cutting surface. First, calculate the area around each point (*a*(*p*) = ∆*X* × ∆*Y*). In the grid, then estimate the area of each slice by multiplying the total number of the points on the grid that hit the slices (∑_*i*=1_^*n*^*p*). Then, the total volume is calculated by multiplying the aggregate areas in slices thickness. Briefly, the total volume of the uterine horn was estimated using the following formulas:

(1) $$\begin{array}{c} V_{\text{total uterine horn}=}\overset{n}{\underset{i=1}{\sum }}p\times a\left(p\right)\times t. \end{array}$$

Volume density of the targeted structure (here perimetrium, myometrium, endometrium, lumen, and uterine gland) was estimated on 5 *μ*m thickness sections through the point-counting method and using Delesse's formula [30]:

(2) $$\begin{array}{c} Vv\left(\text{structure}\right)=\overset{n}{\underset{i=1}{\sum }}p\;\left(\text{structure}\right)/\overset{n}{\underset{i=1}{\sum }}\left(\text{reference}\right). \end{array}$$

“∑_*i*=1_^*n*^*p*(structure)” was the number of the test points falling on the targeted structure (here perimetrium, myometrium, endometrium, lumen, and uterine gland) and “∑_*i*=1_^*n*^*p* (reference)” was the total points hitting the uterine horn sections. The following formula was used to estimate the absolute targeted structure volume [31]:

(3) $$\begin{array}{c} V\left(\text{structure}\right)=V\left(\text{total uterine horn}\right)\times Vv\left(\text{structure}\right). \end{array}$$

#### 2.9.1. Estimation of the Different Layer's Thickness of the Uterine Horn

To evaluate, the mean thickness of the different layers thickness of the uterine horn, an average of 8-12 sections from 5 *μ*m thick sections was randomly selected and studied using the Nikon microscope (e200, Japanese) with a ×100 magnification. To determine measurement sites, the specific line grid (4 parallel lines) was randomly superimposed on the sampled fields. To calculate the mean thickness of the perimetrium, myometrium, and endometrium, the orthogonal intercept method was used. The specific line grid (four parallel lines) was randomly superimposed on the sampled fields. The length of a perpendicular line extending from the inner layer to the outer layer of the uterine horn at each intercept of the line of the grid with the outer layer was considered the orthogonal intercept. An average of 100-200 measurements was estimated and the harmonic mean thickness was calculated using the following formula:

(4) $$\begin{array}{c} \text{zona pellucida mean thickness}=\frac{8}{3\pi }\times \text{number of measurements}/\left(\frac{1}{{oi}_{1}}+\frac{1}{{oi}_{2}}+\frac{1}{{oi}_{3}}+\cdots \right). \end{array}$$

Orthogonal intercepts: number of measurements.

### 2.10. Histopathological Assessment

Hysterectomy was performed and kept in formalin further. H&E slides were performed from each specimen and were analyzed by blind-sided pathologist.

### 2.11. Statistical Analysis

The data obtained from all experimental groups were expressed as mean ± standard error of the mean. Statistical analysis was performed using SPSS for Windows (version 17.0, SPSS Inc., Chicago, IL, USA). Data obtained from *in vivo* multiple groups were compared by one-way analysis of variance (ANOVA) followed by an LSD multiple comparison test and the significance level was set as *p* ≤ 0.05.

## 3. Results

### 3.1. Determination of TPC

The TPC in the 80% hydroethanolic extract was calculated from the equation of the calibration curve of gallic acid extract (GAE). Results showed that the extract contains 46.68 mg total phenol/g dry extract.

### 3.2. Determination of DPPH

The results of the antioxidant assay indicated an IC_50_ value of IC_50_ = 0.463 ± 0.037 mg/ml. The high antioxidant potential of the hydroethanolic extract of licorice root could be due to the presence of a wide variety of bioactive compounds especially phenolics in this plant. Quercetin as positive control demonstrated an IC_50_ value of 4.62 ± 2.26 *μ*M.

### 3.3. Calcium Levels

As depicted in Figure 1, the mean serum calcium levels in the control group were 12.89 mg/dl and there were no significant differences between Sham (Ca level =12.74 mg/dl) and Gly 30% (Ca level =12.71 mg/dl) groups. After OVX, the Ca amount was significantly reduced to 6.51 mg/dl. Interestingly, the Ca level significantly increase in both OVX-Gly 10% and OVX-Gly 30% groups compared to the OVX rat group (*p* < 0.001). The most significant therapeutic effect was seen in OVX-Gly 30% groups (mean =11.71 mg/dl) with no significant differences from the healthy control group.

### 3.4. Alkaline Phosphatase Levels

The ALP levels are presented in Figure 2. It was determined that ALP levels (mean =619.00 IU/l) were significantly higher in the OVX group compared to the control (mean =158.83 IU/l) and Sham group (mean =161.00 IU/l) with *p*-value<0.001. A significant decrease in the ALP levels was observed in the hydroalcoholic extract of licorice root–treated rats compared to the OVX group (*p* ≤ 0.001). In detail, the 30% of licorice root hydroalcoholic extract administration (OVX + Gly 30% group) brought even more decrease in the ALP levels compared to the Gly 10% group.

### 3.5. Estradiol Levels

A significant decrease in plasma estrogen level in the OVX group (mean =5.26 Pmol/l) when compared to the control (mean =22.41 Pmol/l) and Sham (mean =22.50 Pmol/l) groups is shown in Figure 3. The amount of estradiol was significantly higher in the 30% of licorice root hydroalcoholic extract group with a mean value of 17.49 Pmol/l compared to the control group with a *p*-value of <0.001 followed by OVX-Gly 10% (mean =11.69 Pmol/l).

### 3.6. Progesterone Levels

Similarly, the levels of progesterone (*p* < 0.001) were significantly decreased in the OVX group compared with the control and Sham groups (Figure 4). However, the level of progesterone in the treatment group with 30% of licorice root hydroalcoholic extract was significantly increased in comparison with the OVX group (*p* < 0.001).

### 3.7. Stereological Study

#### 3.7.1. Effect of Different Treatments on Perimetrium Thickness and Volume

Data in Figure 5 shows that the perimetrium thickness was reduced by ovariectomy; however, the intake of hydroalcoholic extract of licorice root (10% or 30%) reversed it to normal conditions (Figure 5(a)). A similar trend is also observed in the case of perimeter ovarian volume (Figure 5(b)); it can be seen that the treatment of rats with hydroalcoholic extract of licorice root (10% or 30%) enhanced the volume with a *p*-value of <0.001 compared to OVX group. Noteworthy, 30% hydroalcoholic extract of licorice root exhibited better results in comparison with 30% hydroalcoholic extract of licorice root with a *p*-value of <0.001.

#### 3.7.2. Endometrial Thickness and Volume Assessments

As can be seen in Figure 6, ovariectomy decreased the endometrial thickness (232.97 *μ*M) and volume (31.67 *μ*M) compared with the control and Sham-operated groups (*p* < 0.001). The administration of hydroalcoholic extract of licorice root (10% or 30%) remarkably improved these parameters with a *p*-value of <0.001 concerning the OVX group. Similarly, 30% hydroalcoholic extract of licorice root tends to increase these parameters to normal conditions in comparison with 10% hydroalcoholic extract.

#### 3.7.3. Myometer Ovarian Thickness and Volume Assessments

A significant increase in the myometer ovarian thickness (177.44 *μ*M) and volume (76.83 *μ*M) was detected in the animals which received 10% or 30% hydroalcoholic extract of licorice root compared to the control (*p* < 0.001) (Figure 7). More specifically, 30% hydroalcoholic extract of licorice root significantly increased the myometer ovarian thickness (291.99 *μ*M) and volume (160.42 *μ*M) compared to the control group with a *p* value less than 0.001.

#### 3.7.4. Perimetrium Thickness and Volume Evaluations

As might be expected, perimetrium thickness (3.84 mm^3^) and volume (2.13 mm^3^) evaluations were decreased in the OVX group. A clear growth of thickness (9.44 mm^3^) and volume (9.14 mm^3^) was observed in treatment groups especially in OVX-Gly 30% group compared to the OVX and other tested groups (Figure 8).

#### 3.7.5. Assessments of Vessel Ovarian Diameter

Based on the data presented in Figure 9, ovariectomy decreased the vessel ovarian diameter significantly compared to the control group (*p* < 0.001). Administration of licorice root (10% or 30%) significantly improved the vessel ovarian diameter compared with the OVX group (*p* < 0.001 compare to other tested groups).

#### 3.7.6. Evaluation of Lumen Volume

It is well known that lumen volume was reduced by ovariectomy and administration of licorice root extracts especially at a 30% increase in the lumen volume with *p* < 0.001 compared to OVX and OVX+Gly 10% (Figure 10.).

#### 3.7.7. Evaluation of Uterine Gland Volume

The rats treated with licorice root extracts in different doses (10% or 30%) showed remarkable improvement in uterine gland volume after eight weeks of treatment compared to the OVX group (*p* < 0.001) (Figure 11).

#### 3.7.8. Evaluation of the Volume of the Uterine Horn

As depicted in Figure 12(a), an increase in the volume of the uterine horn was evident in the OVX + Gly 10% and the OVX + Gly 30% groups in comparison to the OVX (*p* < 0.001). However, there are still significant differences in all treated groups compared to Con, Sham, and Gly 30% groups.

### 3.8. Histopathological Study

As mentioned before in “Materials and Methods,” cases were categorized into 6 groups and histopathological findings were evaluated in all groups according to differences between control and other ones. As depicted in Figure 13, in the ovariectomy group, there was a morphologic sign of severe atrophy compared to both Sham and Gly 30% receiving groups. On the other hand, OVX + Gly 10% and OVX + Gly 30% groups showed morphologic evidence of improvement in endometrial and myometrial thickness as well as an increase in the volume of the uterus and the thickness of the layers and glands (arrow mark). There were no significant changes in the Sham group compared to the control group.

## 4. Discussion

Aging is a natural phenomenon associated with a loss of sex hormones in women (menopause) [32]. It would be important to note that during the first year of menopause, women lose around 80% per year of their estrogens. Statistical analysis showed that approximately one in eight women above the age of 55 years has undergone oophorectomy before reaching natural menopause and lost steroidal hormone [33].

Endogenous estrogen deficiency alters biochemical factors including ALP and calcium levels which could be associated with osteoporosis and cardiovascular disease [34]. It is well described that estrogen discrimination declines muscle mass and intensifies the risk for periodontal breakdown, psychiatric symptoms, and impaired sexual functions [35]. The current medication to limit menopause complications and post-oophorectomy problems is estrogen therapy which relieves unpleasant symptoms. On the contrary, estrogen therapy may be associated with an increased risk of breast cancer [36], ovarian cancer [37], endometrial cancer [38], gallbladder disease [39] plus increased overall body fat, central adiposity, and psychiatric symptoms [40, 41]. Considering the health concerns associated with traditional hormone therapy (HT), women seek alternatives to improve their health and relieve menopausal symptoms. Therefore, it is needed a holistic approach to address the problem through the identification and consumption of safe plant-derived estrogens (phytoestrogens).

Phytoestrogens might act as natural selective estrogen receptor modulators, tweaking estrogenic responses in the cardiovascular system, bone, and brain, but dampening responses in the breast and uterus [42]. Also, it has positive impacts on weight loss, skin health, and the immune system. Four phenolic compounds classified as phytoestrogens are Isoflavones, Stilbene, Coumestan, and Lignin [43]. Since ancient times, the root of *Glycyrrhiza glabra* named licorice, as a high source of phytoestrogens, has been known to have a wide range of clinical applications in gastrointestinal disorders (*H. pylori* and peptic ulcer), oral disease, liver disorders, hepatitis B, and hepatitis C and as well as on metabolic disorders. Also, in most cases, phytoestrogens are powerful antioxidants through hydrogen/electron donation and inhibit the development of coronary heart disease and cancers [44, 45].

Data gained in the 2020s reveal that licorice improves bone metabolism. Further evaluation demonstrated this plant inhibits RANKL-induced expression of Nfatc-1, c-Fos, Trap, Ds-stamp, and Ctsk in RAW264.7 cells. Also, fewer amount of bone resorption pits forms when bone marrow-derived monocytes expose to licorice [46]. Another study conducted by Menati et al. on 60 menopausal women was randomly allocated to licorice or hormone replacement therapy (HRT) groups. Results showed that licorice seems more effective than HRT in improving hot flash duration [47]. Similar results were recorded in another study demonstrating that administration of this harmless, inexpensive herb decreased the frequency and severity of hot flashes [48]. Molecular and physiological effects of licorice root administered to ovariectomized mice revealed that licorice reduces body weight gain, overall fat deposition, liver steatosis, and expression of hepatic lipid synthesis genes [49]. Licorice has recently been shown to induce considerable benefits on healthspan and lifespan in middle-aged and older women [50].

It would be interesting to note that the biological and pharmacological properties of medicinal plant constituents are related to structural similarity to metabolites and substrates present in human and animal organisms [51, 52]. Licorice encompasses valuable constituents including Glycyrrhizic acid and Glabridin as well as lots of phenolic and flavonoid constituents [15, 16, 53]. In this case, licorice's main compound has a high structural similarity to steroidal hormones including estrone (E1), estradiol (E2), and estriol (E3) (the structure is presented in Figure 14). These phytoestrogens are usually metabolically active that are converted to enterodiol and enterolactone by the intestinal flora and can be absorbed easily [54, 55]. However, the exact mechanism of action for menopausal was unambiguously established at this time.

In detail, Glycyrrhizic acid is known for steroid-like properties with excellent pharmacological effects such as anti-inflammatory, anti-gastric ulcer, anti-hepatotoxic, and antivirus activities [56]. Treatment with Glycyrrhizic acid and Glabridin increases the organic substances in the femoral bone by 15.3% (*p* < 0.001) [57]. In another study, the favorable effect of Glycyrrhizic acid in the mechanical and histomorphological parameters in the femoral bone was observed. Also, a reduction in serum concentration of Pyridinoline as a bone resorption marker was observed. It was demonstrated that Glycyrrhizic acid may prevent glucocorticoid-induced osteoporosis in rats, by activation of the 11b-hydroxysteroid dehydrogenase enzyme [58].

Glycyrrhizic acid as an aglycone molecule was produced in intestinal flora *via* hydrolyzation of Glycyrrhizic acid. Preliminary data showed that 2 months of Glycyrrhizic acid administration reduced body fat mass by 1% in men and 2.8% in women [59]. It was concluded that Glycyrrhizic acid inhibits 11-*β*-hydroxysteroid dehydrogenase plus suppressing renin activity, improving blood glucose control, and performing a range of corticosteroid-like activities [60].

Glabridin is extensively consumed as an herbal medicine with antioxidant, antiproliferative, and antibreast cancer activities [61, 62]. Glabridin enhanced the function of the osteoblasts cell line [63]. The inhibition of PGE2 and NO production, as well as prevention of osteoblasts apoptosis induced by TNF-a, was observed. This favorable effect of Glabridin could be due to ER-mediated, associated with cellular protection against oxidative stress [63, 64].

Overall, there are two species of nuclear estrogen receptors (ERs) named ER*α* and ER*β* that the configuration of the dimeric nuclear receptor altered following *via* binding to sex steroids [65]. Phytoestrogens can bind to either ER*α* or ER*β* leading to gene expression repression [66]. Phytoestrogens display agonist activity towards the cell surface G-protein coupled estrogen receptor (GPER), as a major mediator of estrogen's rapid cellular effects throughout the body [67]. The mentioned complex binds directly to sex steroid response elements on DNA or indirectly through protein-protein interactions to other DNA sequences such as the AP-1 or SP-1 sites allowing this complex to associate with various intracellular coregulator proteins. However, further research to target this chronic disease is highly needed.

There is still no single best way to reduce the side effect of postmenopausal in OVX women. We have postulated that the lack of beneficial effects of estrogen may compensate with the hydroalcoholic extract of licorice root containing phytoestrogens with estrogen-like properties. In our present study, it was illustrated that licorice increased the Ca and reduced the ALP levels. Also, significant improvement in stereological and histopathological evaluation of uterine tissue was observed.

## 5. Conclusions

Despite the collective evidence outlined, a possible new application of licorice as the traditional plant to the amelioration of postmenopausal undesirable effects and OVX complications, which is becoming a serious problem in women's health care in all society, was identified. Hydroalcoholic extract of licorice root due to containing high amounts of phytoestrogens with similar chemical structures to estradiol notably improves biochemical parameters as well as stereological and histopathological markers of uterine tissues in ovariectomy rats.

## Figures and Tables

**Figure 1:** Effects of ovariectomy and hydroalcoholic extract of licorice root (10% or 30%) on calcium levels in different groups.

**Figure 2:** Effects of ovariectomy and hydroalcoholic extract of licorice root (10% or 30%) on ALP in different groups.

**Figure 3:** Effects of ovariectomy and hydroalcoholic extract of licorice root (10% or 30%) on estradiol levels in different groups.

**Figure 4:** Effects of ovariectomy and hydroalcoholic extract of licorice root (10% or 30%) on progesterone levels in different groups.

**Figure 5:** Effects of ovariectomy and hydroalcoholic extract of licorice root (10% or 30%) on perimetrium ovarian thickness and volume in different groups.

**Figure 6:** Effects of ovariectomy and hydroalcoholic extract of licorice root (10% or 30%) on endometrial thickness and volume in different groups.

**Figure 7:** Effects of ovariectomy and hydroalcoholic extract of licorice root (10% or 30%) on myometer ovarian thickness and volume in different groups.

**Figure 8:** Effects of ovariectomy and hydroalcoholic extract of licorice root (10% or 30%) on perimetrium thickness and volume in different groups.

**Figure 9:** Effects of ovariectomy and hydroalcoholic extract of licorice root (10% or 30%) on vessel ovarian diameter in different groups.

**Figure 10:** Effects of ovariectomy and hydroalcoholic extract of licorice root (10% or 30%) on lumen volume in different groups.

**Figure 11:** Effects of ovariectomy and hydroalcoholic extract of licorice root (10% or 30%) on uterine gland volume in different groups.

**Figure 12:** Effects of ovariectomy and hydroalcoholic extract of licorice root (10% or 30%) on the volume of uterine horn in different groups.

**Figure 13:** Histopathological study of uterus tissue and the effect of treatments in uterus tissues in ovariectomized rats. (a) Control group. (b) Sham group. (c) Gly 30% group. (d) OVX. (e) OVX + Gly 10%. (f) OVX + Gly 30%.

**Figure 14:** Chemical structure of steroidal hormones and major licorice constituents.

## Data Availability

All data generated or analyzed during this study are included in the manuscript.
